# Randomized Controlled Study of the Effects of DHEA on the Outcome of IVF in Endometriosis

**DOI:** 10.1155/2021/3569697

**Published:** 2021-10-14

**Authors:** Yanxia Zhang, Meiqing Li, Lian Li, Jianghua Xiao, Zhe Chen

**Affiliations:** ^1^The Second Affiliated Hospital, Department of Reproductive Center, Hengyang Medical School, University of South China, Hengyang, Hunan 421001, China; ^2^The Second Affiliated Hospital, Department of Respiratory, Hengyang Medical School, University of South China, Hengyang, Hunan 421001, China

## Abstract

**Objective:**

To investigate the effect of dehydroepiandrosterone (DHEA) on the outcome of in vitro fertilization (IVF) in patients with endometriosis (EMT).

**Methods:**

Female patients diagnosed with EMT in our hospital from May 2018 to May 2019 were selected. The patients were divided into the control group (*n* = 22) and the DHEA group (*n* = 22) according to the random number table. Patients in the control group received placebo and patients in the DHEA group received DHEA. Patients in both groups received either DHEA (25 mg) or placebo orally 3 times a day for 90 days from the first day of menstruation. Patients were subsequently treated with an IVF cycle. In the control group, 22 patients completed the first cycle and 13 patients completed the second cycle. In the DHEA group, 22 patients completed the first cycle and 11 patients completed the second cycle. Serum sex hormone levels including serum E2 on hCG day, mean progesterone on hCG day, FSH on day 2, AMH on day 2, and gonadotropin dose were determined using a chemiluminescent immunoassay kit. The number of antral follicles of the bilateral ovaries was counted by transvaginal B-ultrasound, and the maximum length and transverse diameter of the ovaries were measured at the same time, to calculate the average diameter of the ovaries, observe the morphology of endometrium, and measure the thickness of the endometrium. The implantation rate, clinical pregnancy rate, persistent pregnancy rate, and live birth rate were compared between the two groups.

**Results:**

There were no significant differences in serum E2, progesterone, endometrial thickness, recovered oocytes, mean number of transferred embryos, and mean score of leading embryo transfer between the DHEA group and the women who completed the first and second cycles (*P* > 0.05). The AMH, antral follicle count, serum E2 on hCG day, the number of recovered oocytes, fertilized oocytes, and the fertilization rate in the DHEA group were higher than those in the control group (*P* < 0.05). The doses of FSH on day 2, COH on day 3, and gonadotropin were lower than those in the control group (*P* < 0.05). There was no significant difference in the total number of embryos, the number of high-quality embryos, and the number of transplanted embryos between the two groups (*P* > 0.05). The implantation rate, clinical pregnancy rate, persistent pregnancy rate, and live birth rate in the DHEA group were higher than those in the control group (*P* < 0.05).

**Conclusion:**

DHEA can significantly increase serum E2 level and improve IVF outcome by regulating the hormone synthesis process, thus improving oocyte and embryo quality.

## 1. Introduction

As a hormone-dependent disease, it is reported that endometriosis (EMT) occurs in 16–50% of infertile women [1, 2]. The causal relationship between EMT and infertility has not been clarified, but it has been assumed that the combination of distorted pelvic anatomy, the immune modulation within the peritoneal cavity, the altered peritoneal function, a diminished ovarian reserve, and an altered endometrial receptivity could be the cause of infertility [3]. In addition, the endometrium of women with endometriosis is resistant to the selective actions of progesterone, which is a hormone that affects decidualization and regulates the local inflammation during implantation [4]. Women with EMT often require in vitro fertilization (IVF) to increase the probability of pregnancy, and more than 1/3 of the women who underwent IVF cycles have been diagnosed as EMT [5]. However, compared with infertility women of other causes, women with EMT always result in poor IVF outcomes for the reduced ovarian response caused by EMT [6]. There are many possible reasons for the poor outcome of IVF, such as the factors of reproductive endocrine, endometrial receptivity abnormality, abnormal embryo implantation, and the failure of embryogenesis and development. At present, many studies focus on the causal relationship between embryo transfer and the poor results of IVF. It is reported that dehydroepiandrosterone (DHEA), which is mainly secreted by the adrenal cortex and ovarian follicle cells, is related to age-related changes in cardiovascular tissues, female fertility, metabolism, and neuron/central nervous system functions [7]. Triantafyllidou et al. [8] used DHEA for the first time on elderly women with a poor ovarian response, which has been proved to be effective in regulating the ovarian response. Since then, more studies have documented the beneficial role of DHEA in modulating the ovarian response, thus improving the IVF outcome [9–12]. It has been proved that a low dose of androgen can promote the recruitment of follicular reserve and enter into the growth and development area of POR patients, and under the action of androgen, both the antral follicle and the androgen receptor on the antral follicle can play a role in promoting the proliferation of follicular membrane cells and granulosa cells. Finally, it leads to the decrease of egg apoptosis and follicular atresia, thus improving the ovarian reserve function (the dual effects of androgen on follicular development). There is no report about the application of DHEA in emergency patients. The purpose of this study is to find out the positive effects of DHEA on women with endometriosis undergoing IVF.

## 2. Materials and Methods

### 2.1. Patients

Select women who were diagnosed with EMT in our hospital from May 2018 to May 2019. Inclusion criteria [13] were as follows: (1) age between 25 and 40 years; (2) women who had tried to conceive for at least 1 year; (3) women who will receive IVF; and (4) women who were diagnosed with EMT. Exclusion criteria [13] were as follows: (1) women who have experienced three or more IVF cycles with no success; (2) women diagnosed with uterine malformation or abnormality; (3) women diagnosed with hydrosalpinx; (4) women who had experienced two or more spontaneous abortions; (5) couples with female or male diagnosed with chromosome abnormality; (6) women who had carried out chemotherapy with cytotoxic agents; (7) women who had carried out pelvic radiotherapy; (8) women who had taken DHEA before the enrollment; (9) women with a history of epilepsy; (10) women with PCOS; and (11) women who are allergic to DHEA.

EMT patients (*n* = 65) who met the study inclusion and exclusion criteria and agreed to join the study were divided into the control group (*n* = 33) (placebo) and the DHEA group (*n* = 32) by random number table method. Before the start of the IVF cycle, 11 patients in the control group withdrew from the study due to pregnancy or personal reasons, and 10 patients in the DHEA group withdrew from the study due to pregnancy or personal reasons. In the end, 22 patients in the control group participated in the study. 22 patients completed the first cycle, and 13 patients example completed the second cycle. In the DHEA group, 22 patients participated in the study, 22 patients completed the first cycle, and 11 patients completed the second cycle. A total of 68 cycles were carried out. The flow of the participants of this study is described in Figure 1.

### 2.2. Research Method

Patients in the control group were treated with placebo, while patients in the DHEA group were treated with DHEA. Two groups of patients took the oral administration of DHEA (25 mg) or placebo three times a day from the first day of the menstrual period for 90 days [14, 15]. Both the DHEA (DHEA, Natrol, USA) and placebo components were prescribed by pharmacists who did not participate in this clinical study. The pharmacist packed the DHEA and placebo pills according to the random list and labeled the subject number on the drug packaging. The participants underwent the IVF cycle afterward.

A long-term IVF-ET protocol was used in this research. On day 2 of menstruation, all women received human menopausal gonadotropin (hMG; Merional1, IBSA, Lugano, Switzerland); the initial dose ranged between 300 and 450 IU per day and was adjusted according to the patient's response guided by the number and size of the follicles as well as the serum E2 levels. When the dominant follicle reached 14 mm, cetrorelix (0.25 mg, Cetrotide® Merck Serono, Darmstadt, Germany) was given daily and COH was continued until at least three follicles grew to 17 mm in size. Afterward, the patients received the administration of 10000IU of human chorionic gonadotrophin (hCG; Choriomon®, IBSA). Oocyte retrieval was guided by transvaginal ultrasound and was performed 34–36 h after hCG administration. The procedure should be cancelled if less than 3 follicles ≥17 mm in size were present 12 days after starting follicle-stimulating hormone (FSH). The decision of either conventional intracytoplasmic sperm injection (ICSI) or in vitro fertilization (IVF) to be performed in each participant was made by the embryologist, which was depending on the recent results of semen analysis and the history of past treatment cycles. Zygotes were then transferred to a global culture medium (Life Global, Ontario, Canada). The embryos that contain 6–8 even blastomeres with <10% fragmentation at day 3 were identified as excellent quality. The embryo transfer was performed on day 5 after the oocyte retrieval, one or two (if possible) embryos were transferred, and the remaining embryos were cryopreserved. Luteal support was given using progesterone vaginal suppository started from the day of oocyte retrieval. Serum *β*-hCG was measured 2 weeks after embryo transfer.

Cycle cancellation criteria were as follows: (1) there are no dominant follicles 7 days after ovulation induction; (2) the dominant follicles show no increase in size for three consecutive days and E2 is observed ass declining; (3) the size of the dominant follicles is less than 14 mm and the endogenous LH surge is observed in the urine or serum; (4) luteinized unruptured follicle syndrome (LUFS) occurs during the process of monitoring; (5) all oocytes failed to be fertilized; and (6) embryos cannot be transferred.

### 2.3. Observation Index

The chemiluminescent immunoassay kit was used to measure the serum sex hormone level, including serum E2 on hCG day, mean progesterone on hCG day, day 2 FSH, day 2 AMH, and gonadotropins doses. The determination of the basic hormones in serum is carried out by the full-automatic electrochemical Luminescent Immunoassay Instrument and the corresponding kit (Beckman, United States).

The number of the antral follicles in bilateral ovaries, that is, basic AFC, was counted by vaginal B-ultrasound. At the same time, the maximum length and transverse diameter of ovary were measured, the average diameter of ovary was calculated, and the shape and the thickness of endometrium were observed. All of the follicular monitoring was carried out by the same experienced doctor.

The clinical pregnancy is defined as the presence of an intrauterine gestational sac 5 weeks after embryo transfer. Continuous pregnancy was defined as fetal heartbeat confirmed by ultrasound at 12 weeks of pregnancy. Implantation rate was calculated by dividing the number of gestational sacs by the total number of transferred embryos. The live birth is newborns (>28 weeks of gestation) who were delivered with signs of life.

## 3. Statistical Method

The results of this experiment were statistically analyzed by SPSS 20.0 (SPSS Co., Ltd., Chicago, USA). Count data were expressed by (rate), and a chi-square test was used for their comparison between groups. Measurement data were expressed by mean ± standard deviation, and *t*-test was used for their comparison between groups. The measurement data that do not obey the normal distribution are represented by the median, and the Mann–Whitney *U* test is used for comparison between groups. *P* < 0.05 indicates that the difference is statistically significant.

## 4. Results

### 4.1. Comparison of General Data Statistics between the Two Groups

There were no statistically significant differences between the two groups in the general data statistics such as average age, body mass index, duration of subfertility, basal FSH, serum E2 on hCG day, mean progesterone on hCG day, retrieved oocytes, and mean number of embryos transferred (*P* > 0.05). The basic conditions of the two groups were similar, and they were comparable as shown in Table 1.

### 4.2. Comparison of the Successive Cycles of the DHEA Group

The explore the cumulative effect of DHEA during the whole study period. The cycle outcomes were compared between the first and second cycles of the women in the DHEA group who had completed the two DHEA treatment cycles. There was no significant difference in serum E2, progesterone, endometrial thickness, number of eggs obtained, average number of transferred embryos, and average score of the first and second embryo transfer between women who received the first and second cycle (*P* > 0.05) as shown in Figure 2.

### 4.3. Comparison of Treatment Cycle between the Two Groups

Day 2 AMH, antral follicle count, serum E2 on hCG day, retrieved oocytes, fertilized oocytes, and fertilized rate in the DHEA group were all higher than those in the control group; the difference was statistically significant (*P* < 0.05). Day 2 FSH, days of COH, and gonadotropins doses were all lower than the control group; the difference was statistically significant (*P* < 0.05). There was no significant difference between the two groups in the total number of embryos, the number of excellent embryos, and the number of transferred embryos (*P* > 0.05) as shown in Table 2.

### 4.4. Comparison of the Effect on In Vitro Fertilization between the Two Groups

In the control group, pregnancy occurred in 3 cycles (8.57%), 2 patients (5.71%) of continuous pregnancy, and 2 patients (5.71%) of live birth. In the DHEA group, there were 8 cycles of pregnancy (24.24%), 7 patients (21.21%) of continuous pregnancy, and 6 patients (18.18%) of live birth. The implantation rate, clinical pregnancy rate, persistent pregnancy rate, and live birth rate in the DHEA group were higher than those in the control group, and the differences were statistically significant (*P* < 0.05) as shown in Table 3.

## 5. Discussion

The infertility rate of patients with endometriosis is significantly higher than that of nonendometriosis, which has attracted the increasing attention of clinical researchers. It is reported that several prognostic factors are associated with infertility caused by endometriosis. The causes of infertility in EMT women may range from anatomical distortions [16] to immunological disorders [17]. Many studies at home and abroad have shown that infertile women often have mild EMT, but it is not clear whether there is an adverse pregnancy outcome after IVF-ET treatment compared with patients without endometriosis. Although the severity of clinical symptoms of EMT may not be directly proportional to the time of infertility and the complexity of treatment of infertility, some studies have confirmed that severe EMT will affect the embryo implantation rate and clinical pregnancy rate of infertile women. Compared with other methods of assisted pregnancy, assisted reproductive technology has a significantly higher success rate and has become an important method for treating infertility in recent years. IVF has become an effective treatment choice in women with EMT; however, the women with more advanced stages of EMT have a lower success rate [18], which may relate to the lower ovarian response compared with the less advanced disease stages. In recent years, low dose androgen has been proved to be beneficial in the treatment of patients with ovarian hyporesponsiveness. It was found that, before or during IVF-ET treatment, the granulosa cells of the ovaries have a higher sensitivity to FSH, which results in an increase in the obtained oocytes and the improved quality of embryos. According to the existing data, oral administration of DHEA and percutaneous administration of testosterone are the two most commonly used methods of androgen supplementation. Since the initial report that documented DHEA has positive effects on ovarian response, embryo quality, and pregnancy outcomes in women receiving IVF [19, 20], a series of clinical trials start to accumulate to verify the benefit of DHEA. However, the use of DHEA in women with EMT has not been investigated.

This research proves that DHEA can improve the IVF outcome in women with EMT-related infertility. Although the sample size is a significant limitation of this study, our findings show a higher pregnancy and live birth proportion of the EMT women in the DHEA group. Our study also documents that the supplement of DHEA in women with EMT can significantly decrease the FSH level, increase the level of AMH and the number of sinus follicles, and significantly improve ovarian function. These results are consistent with the beneficial effect of DHEA in previous reports.

DHEA, a mild androgen, is a precursor of E2 and testosterone and serves as an important prehormone of sex steroidogenesis. The levels of the DHEA cycle decreased significantly with the increase of age [21]. Casson [8] reported for the first time that exogenous DHEA supplementation could restore follicular steroid production in the ovaries of elderly women. Although DHEA has positive effects in improving the ovarian response, the mechanisms underwent are still unclear. In the research aimed at clarifying how DHEA affects infertility, many assumptions have been established. The ovarian folliculogenesis, for instance, is hypothesized to be directly affected by DHEA, and the primordial follicle pool was then increased up to the preantral and antral follicle stages [22]. Androgens may affect ovarian follicular development by regulating the amount of FSH receptors that are expressed in the granulosa cells [23], and the increased intrafollicular androgens could stimulate the granulosa cell to produce more AMH [14], thus promoting the early stages of follicular growth [8]. An animal model research has proved that the supplement of DHEA could promote the proliferation of the granulosa cell and then stimulate the initiation of primordial follicles and the development of gonadotrophin-responsive preantral and early antral follicles [22]. In addition, oral DHEA supplement has been proved to upregulate the concentration of IGF-1 in serum [24], which is well known, and has a beneficial effect on follicular development and oocyte quality. This indicates that the positive effect of DHEA may be modulated by the increase of IGF-1. IGF-1 has been known to have synergistic effects on FSH and then increase the effect of FSH on E2 and progesterone secretion. Moreover, IGF-1 is also an important factor for the maturation of oocytes. Furthermore, DHEA may also improve the follicular microenvironment by decreasing the apoptosis of the originally recruited follicles and ameliorating the function of mitochondrial in both follicular cells and oocytes [25]. In addition, given the proof that DHEA can reduce the miscarriage rate in elderly women [26], which may benefit from the decreased aneuploid embryo rates [27], DHEM may improve the quality of oocyte by promoting DNA repair in oocytes [28].

The level of follicle-stimulating hormone in the DHEA group decreased significantly, which indicated that DHEA supplementation improved ovarian reversal. There are many indexes in the evaluation of ovarian reserve function, but the most common and convenient one is the basic follicle-stimulating hormone (bFSH) level on the 2^nd^-3^rd^ day of the menstrual cycle. The number of follicles decreases in patients with low ovarian reserve, which greatly reduces the sensitivity of follicles to FSH, thus affecting the growth and development of follicles. The continuous high expression of follicle-stimulating hormone severely inhibits the function of follicles, which is due to the fact that the excessive follicle-stimulating hormone can increase the release of the gonadotropin-releasing hormone through the action of the hypothalamic-pituitary-ovarian axis under the positive feedback, thereby further improving the level of follicle-stimulating hormone and finally leading to the occurrence of adverse ovarian reactions. The reduction of FSH caused by DHEA might contribute to its stimulation on the anterior follicle and the androgen receptors above; thus, the stromal cells and granulosa cells of the follicle membrane were promoted to proliferate.

This study also suggested that DHEA can increase the number of follicles in the basal sinus. The antral follicles (AFC) are the precursor of maturity, of which the diameter is less than 10 mm. With the development of follicles, AMH expression was the highest in 2–8 mm preantral follicles and small antral follicles, but the secretion of AMH stopped at the 8–10 mm FSH dependent stage. DHEA increased the number of antral follicles, thus increasing the AMH secretion and the level of AMH in serum.

Taken together, this is evidence to clarify that DHEA has beneficial effects on the IVF outcome in women with EMT. DHEA pretreatment significantly increased the serum level of E2, suggesting that DHEA may improve IVF outcome by modulating the process of hormone synthesis and then improve the quality of oocyte and embryo. We have realized that the sample size could be a weakness of this study. However, considering that women with endometriosis suffer from infertility and are unwilling to “waste” their time taking the placebo, the possibility of the selection deviation might be limited. A larger multicenter trial is needed to enhance the results of this study.

## 6. Conclusion

EMT may cause infertility throughout a broad range of mechanisms, including peritoneal inflammation and endocrine disorders, which interfere with ovarian response and finally reduce oocyte competence. Our analysis suggests that DHEA may play an essential role in improving the ovarian response, thus ameliorating the IVF outcome in women with EMT.

## Figures and Tables

**Figure 1:** Study flowchart.

**Figure 2:** Comparison between the two successive cycles of the study group.

**Table 1:** General data statistics of the two groups.

	Control group (*n* = 22)	DHEA group (*n* = 22)	*t*	*P*
Average age (years)	37.46 ± 2.17	38.61 ± 2.93	1.479	0.146
Body mass index (kg/m^2^)	24.53 ± 0.69	24.16 ± 0.86	1.574	0.123
Duration of subfertility (years)	7.64 ± 0.41	7.82 ± 0.29	1.867	0.069
Basal FSH (IU/ml)	8.76 ± 2.13	8.93 ± 2.57	0.239	0.812
Serum E2 on hCG day (pg/mL)	1456.82 ± 594.28	1629.43 ± 615.74	0.946	0.349
Mean progesterone on hCG day (ng/mL)	0.59 ± 0.21	0.61 ± 0.28	0.268	0.790
Retrieved oocytes (pieces)	5.98 ± 0.34	6.21 ± 0.45	1.913	0.063
Mean no. of embryos transferred (pieces)	1.28 ± 0.42	1.46 ± 0.51	1.278	0.208

**Table 2:** Comparison of treatment cycle between the two groups and the effect on in vitro fertilization (*n* (%), mean ± SD).

	DHEA group cycles (*n* = 33)	Control group cycles (*n* = 35)	*t/Z*	*P*
Day 2 FSH (IU/ml)	11.82 ± 0.92	9.25 ± 0.97	11.213	≤0.01
Day 2 AMH (ng/mL)	0.84 ± 0.22	1.35 ± 0.19	10.203	≤0.01
Antral follicle count	7.63 ± 1.92	9.75 ± 0.38	6.226	≤0.01
Serum E2 on hCG day (pg/mL)	1303.61 ± 591.72	1598.94 ± 612.15	2.023	0.047
Retrieved oocytes (pieces)	5.91 ± 0.35	6.98 ± 3.14	2.004	0.049
Fertilized oocytes (pieces)	3.70 ± 1.71	4.69 ± 2.24	2.056	0.044
Fertilized rate (%)	50.13 ± 29.12	65.39 ± 27.31	2.226	0.030
Days of COH (days)	12.92 ± 2.37	11.26 ± 2.91	2.586	0.013
Gonadotropins doses (IU)	3952.73 ± 871.16	3541.87 ± 729.25	2.102	0.039
Total number of embryos (pieces)	2.5 (0–7)	2.7 (0–8)	−1.085	0.346
Number of excellent embryos (pieces)	1 (0–4)	2 (0–5)	−1.168	0.329
Number of transferred embryos (pieces)	1.59 ± 0.51	1.82 ± 0.46	1.949	0.056

**Table 3:** Comparison of the effect on in vitro fertilization between the two groups (*n* (%)).

	DHEA group cycles (*n* = 33)	Control group cycles (*n* = 35)	*χ* ^*2*^ */Z*	*P*
Implantation rate	0 (0–0.5)	0 (0–1)	−2.608	0.012
Clinical pregnancy	3 (8.57%)	8 (24.24%)	3.264	0.019
Ongoing pregnancy	2 (5.71%)	7 (21.21%)	2.194	0.032
Live birth	2 (5.71%)	6 (18.18%)	2.375	0.026

## Data Availability

The data can be obtained from all the authors upon reasonable request.
